The article "A Hybrid Genetic Algorithm for Nurse Scheduling Problem considering the Fatigue Factor" was published in 2021. Journal: J Healthc Eng.

# A Hybrid Genetic Algorithm for Nurse Scheduling Problem considering the Fatigue Factor

**DOI:** 10.1155/2021/5563651

**Published:** 2021-03-31

**Authors:** Atefeh Amindoust, Milad Asadpour, Samineh Shirmohammadi

**Affiliations:** ^1^Department of Industrial Engineering, Najafabad Branch, Islamic Azad University, Najafabad, Iran; ^2^Department of Information Systems and Operations Management, Business School, The University of Auckland, Auckland, New Zealand; ^3^Young Researchers and Elite Club, Najafabad Branch, Islamic Azad University, Najafabad, Iran

## Abstract

Nowadays and due to the pandemic of COVID-19, nurses are working under the highest pressure benevolently all over the world. This urgent situation can cause more fatigue for nurses who are responsible for taking care of COVID-19 patients 24 hours a day. Therefore, nurse scheduling should be modified with respect to this new situation. The purpose of the present research is to propose a new mathematical model for Nurse Scheduling Problem (NSP) considering the fatigue factor. To solve the proposed model, a hybrid Genetic Algorithm (GA) has been developed to provide a nurse schedule for all three shifts of a day. To validate the proposed approach, a randomly generated problem has been solved. In addition, to show the applicability of the proposed approach in real situations, the model has been solved for a real case study, a department in one of the hospitals in Esfahan, Iran, where COVID-19 patients are hospitalized. Consequently, a nurse schedule for May has been provided applying the proposed model, and the results approve its superiority in comparison with the manual schedule that is currently used in the department. To the best of our knowledge, it is the first study in which the proposed model takes the fatigue of nurses into account and provides a schedule based on it.

## 1. Introduction

In working places such as hospitals where the services must be provided continuously, distribution of workforces within different shifts is required. Accordingly, different studies could be found within the literature which formulated the problem of scheduling nurses, known as the Nurse Scheduling Problem (NSP), from different aspects to provide a timetable for nurses in a hospital [1–3].

In NSP, nurses are assigned different shifts according to a set of constraints and requirements which are determined by the hospital. On one hand, optimal nurse scheduling has effects on reducing hospital costs, increasing nurse's job satisfaction, quality of care, and increasing the input budget of hospitals [4]. On the other hand, hospital work shifts could impose negative effects on involved nurses such as understaffing, heavy workload, and irregular work-scheduling conditions. It adversely affects the service quality of healthcare operations and leads to less patient-nurse interaction and patient safety issues. Meanwhile, other negative impacts of shift works on nurses are important such as fatigue, obesity, sleep disorder, and a wide range of chronic diseases [5–8]. It seems that human factors should be combined with NSP if a more productive hospital is needed. In other words, studying NSP considering human factors could improve both the performance of nurses and productivity of hospitals significantly [9].

In addition to former issues in nurses' work shifts, the pandemic of the COVID-19 has aggravated the problem and put double pressure on nurses across the world. In this new situation, work shifts should be determined regarding response to patients' care requirements effectively and immediately and reduction of nurses' fatigue simultaneously.

Motivated by the aforementioned issues, and since, to the best of our knowledge, formulating an NSP considering fatigue factor has not studied yet, in this study, we have suggested a framework to distribute nurses in work shifts with the least fatigue alongside an attention to the additional pressure due to COVID-19 pandemic. To do so, a mathematical model is formulated for NSP in which fatigue of nurses has been taken into account. To solve the proposed model, a hybrid Genetic Algorithm (GA) has been developed, and real data from a department in one of the hospitals in Esfahan, Iran, where COVID-19 patients are hospitalized, has been used to provide a timetable for May.

The remaining parts of the current paper are as follows.

Firstly, related previous work on the area of NSP is investigated. After that, the problem is described and formulated, and then, the proposed GA is introduced. Following this, test problems are solved to approve the accuracy of the proposed model. Next, a real case study is considered, and a timetable for the department of COVID-19 patients is provided. Also, results are compared with the current timetable which is scheduled manually. Finally, the most important results along with suggestions for future research are presented in the conclusion section.

## 2. Literature Review

Taking preferences into account has been studied in NSP from different points of view. For instance, in the NSP study of Tsai and Li [10], Topaloglu and Selim [11], Abdollahi and Ansari [12], Wong et al. [13], Jafari et al. [14], and Legrain et al. [15], shift preferences were considered while in Vanhoucke and Maenhout [16] both shift preferences and day preferences were integrated simultaneously. Also, Liu et al. [17] considered NSP in hemodialysis service with a preference on roles and shifts. Further, Hamid et al. [9] proposed a multiobjective model for NSP considering the skill, preference, and compatibility of nurses.

In addition to preferences, some papers have added social/human factors into the NSPs. For example, in Farasat and Nikolaev [18], social structure effects into Nurse Scheduling Problem (NSP) were considered, and it was shown how the social structure of the working environment can affect the performance of nurses. In Zanda et al. [19], the maternity of nurses, type of their contracts (full time or part time), or nurses that benefit from special reductions of the workload for several reasons (e.g., because they have a close relative who suffers a serious illness) have been taken into account in providing a nurse schedule. Nahand et al. [20] proposed a multiobjective model for NSP considering human errors of nurses to determine optimal shift scheduling of nurses. Particularly, nurses' preference score, allocation costs, penalty cost of violating soft constraints, and human errors were all considered as objectives to be optimized, and a weighted-sum method was employed to solve the model. Wolbeck et al. [21] proposed a model for the NSP considering the timing and distribution of shift changes among nurses. In fact, the model incorporates a fair shift change penalization scheme, in which the type, timing, and distribution of shift changes among nurses are taken into account. In addition, information from previous periods was considered, using an individual penalty score to distribute the shift changes fairly among the nurses. The model was solved within the Gurobi software.

Assigning nurses to the operating room is the subject of another group of papers in the NSP literature. Lim et al. [22] presented two models for NSP. The first one assigns nurses to upcoming surgery cases while the second one assigns lunch breaks for nurses. A column generation algorithm and a two-phase swapping heuristic were developed to find feasible assignments in a fast manner. In another study, Di Martinelly and Meskens [23] proposed a biobjective model for NSP to assign nurses to operating rooms. They have used the *e*-constraint method to solve the problem. Besides, Chiang et al. [24] presented a mathematical model which can provide an optimized schedule for nurses and operating rooms simultaneously. GAMS software was deployed to solve the proposed model.

Also, categorizing patients into different groups and then assigning nurses to each group of them have been studied in NSPs as well. In particular, Heshmat et al. [25] studied a two-stage approach where, at the first stage, patients are clustered, and then, at the second stage, nurses are assigned to each cluster. The model was solved by using CPLEX. Moreover, Sarkar et al. [26] proposed a framework to assign nurses to home patients and patients in the hospital according to different demands with respect to the patients' health status. A hybrid GA was applied to solve the problem.

Meanwhile, the possibility of exchanging nurses within different departments has also been investigated. Fügener et al. [27] proposed a mid-term model for NSP considering cross-training effects. Firstly, a framework to define and visualize cross-training policies was proposed. Next, a new cross-training policy was introduced where each unit trained one dedicated nurse for each other unit, and finally, by using *g* CPLEX for solving the model, a schedule was provided. He et al. [28] proposed a two-stage stochastic model for NSP considering understaffing risk control. In the proposed model, an initial base number of nurses within the department's budget were assigned to the department. However, a central pool of nurses was maintained from where extra nurse shifts can be transferred from the pool to cover the shortage in certain departments, or redundant nurse shifts can be transferred into the pool. The model was solved using CPLEX. Schoenfelder et al. [29] presented a model that incorporates two classes of quick-response decisions in hospitals' nurse scheduling, namely, adjustments to the unit assignments of cross-trained float nurses and transfers of patients between units and off-unit admissions. They have examined the proposed model within different hospitals.

However, the main purpose of some papers is to develop heuristic/metaheuristic/simulation-based approaches for solving NSPs with the aim of improving the solution procedures from both quality and CPU time. In this case, hybrid Artificial Bee Colony (Awadallah et al. [30]), Particle Swarm Optimization (Wu et al. [31]), Sample Average Approximation method (Bagheri et al. [32]), Variable Neighborhood Search algorithm (Zheng et al. [33], Rahimian et al. [34]), Hybrid Harmony Search algorithm (Awadallah et al. [35]), a heuristic approach based on Simulated Annealing (Knust and Xie [36]), a combination of three algorithms, namely, Fix-and-Relax, Fix-and-Optimize, and Simulated Annealing (Turhan and Bilgen [37]), and a heuristic procedure based on column generation (Strandmark et al. [38]) could be found within the literature of NSP.

According to a comprehensive literature review, we did not find any research which formulated NSP considering fatigue factor. To fill this research gap and to decrease double pressure which has been imposed on nurses due to the spreading of COVID-19, in the current paper, we formulated the NSP by considering the fatigue factor for a real case study, a department in one of the hospitals in Esfahan, Iran, where COVID-19 patients are hospitalized, to provide a schedule for nurses of this department for May in all shifts.

## 3. Problem Description

Health organizations such as hospitals are responsible for providing required services in both normal and crisis situations [39–41]. In recent years, health management has received special attention among researchers since appropriate allocation and usage of resources are vital to provide high-quality services to patients [42]. Accordingly, researchers in conjunction with decision-makers have worked on health management (as a pivotal issue in many political and social debates) in different regions and countries across the world to select an optimal form for the usage of healthcare resources [43]. To do so, they have applied novel decision-making tools to allocate and productive usage of resources [44] since the quality of the provided services to patients is highly dependent on the available resources. Among required resources, human resources are the most important factor in providing services [45, 46]. Because staff costs are a heavy part of each organization's cost, increasing the productivity and efficiency of human resources is very significant. One of the most practical ways to increase the productivity of this valuable resource is to combine the right distribution of human resources [47, 48]. In other words, it is very important to determine the number of required nurses during each shift so that, depending on the volume of arrivals, the provision of services always remains at the desired level. There are different types of shifts such as night shifts, last week shifts, two-part shifts, and on-call shifts. However, work shifts should be scheduled in such a way that imposes the lowest fatigue on nurses because long shifts have a negative efficacy on employee physiology. To do so, we propose a multiobjective model for the Nurse Scheduling Problem to optimize the work shifts of nurses, which includes three shifts in the morning, evening, and night. The first objective function is minimizing the total costs while the second objective function is minimizing the expected value of total fatigue for all nurses in all shifts. In fact, in this model, since fatigue is one of the main human factors which affects the quality of doing jobs and health circumstances of employees, the nurse fatigue factor has been investigated as a function with binary values according to break times which makes a virtual life for nurses. In simple words, to reduce nurses' fatigue during the shifts, some certain times are allocated for their break.

Some of the assumptions of the problem are as follows:

- All nurses have identical skills
- The break times are discrete values
- Demand behavior is the random variable based on a specific distribution function
- Each nurse is only assigned one shift
- The break time is more important compared with shift time

### 3.1. Sets and Parameters

 
*i*: Period (day)
 
*j*: Rest time (break time)
 
*c*_1_: Employment cost
   *c*_2_: Dismissal cost
 
*c*_3_: Nurse shortage cost
 
*c*_4_: Nurse surplus cost
 
*c*_5_: Fatigue reduction cost
 
*τ*_*ij*_: Duration of the rest time *j* at period i
   *L*_*i*_: Duration of the shift time at period i
 
Δ_*i*_: Interval between the breaks at period i
 
*b*: Maximum fatigue level
 
*a*: positive value
 
*γ*: positive value
 
*P*: A very large number

### 3.2. Decision Variables and Functions

 
*x*_*i*_: Nurse level changes at period i
 
*m*: Rest level (integer positive values use for determining rest time)
 
*D*: Required nurse number
 
*v*_*ij*_: Nursing attendance virtual time based on rest time *j* at period i
 
*f*(*d*): Probability function of required nurse number
 
*F*(*t*): Fatigue function
 
*δ*(*m*): Fatigue fix function
 
*c*_*PM*_(*i*): Nurses' fatigue reduction function at period i
 
*W*: A binary variable, which is equal to 1 if nurse's employment is required; 0, otherwise
 
*Z*: A binary variable, which is equal to 1 if nurse's dismissal is required; 0, otherwise

### 3.3. Model Formulation

(1) $$\begin{array}{c} \min f_{1}=\overset{T}{\underset{i=1}{\sum }}c_{PM}\left(i\right)+c_{1}\overset{T}{\underset{i=1}{\sum }}x_{i}^{+}+c_{2}\overset{T}{\underset{i=1}{\sum }}x_{i}^{-}+c_{3}\overset{T}{\underset{i=1}{\sum }}\overset{D_{\max}}{\underset{D=x_{i}}{\sum }}\left(D-x_{i}\right)\frac{e^{-\lambda t}.\lambda t^{D}}{D!}\;+c_{4}\sum_{i=1}^{T}\sum_{D=x_{i}}^{D_{\max}}\left(x_{i}-D\right)\frac{e^{-\lambda t}.\lambda t^{D}}{D!}, \end{array}$$

(2) $$\begin{array}{c} \min f2=\sum_{i=1}^{T}x_{i}\left[\int_{0}^{\tau_{i1}}F\left(t\right)\text{d}t\;+\sum_{j=2}^{n}\int_{\tau_{ij-1}}^{\tau_{ij}}F\;\left(v_{ij}+t-\tau_{ij-1}\right)\text{ d}t+\int_{\tau_{ij-1}}^{L_{i}}F\left(v_{in}\;+t-\tau_{in}\right)\text{ d}t\right] \end{array}$$

subject to

(3) $$\begin{array}{c} v_{ij}=v_{ij-1}+\delta \left(m\right)\cdot \left(\tau_{ij}-\;\tau_{ij-1}\right)\;i=1,\ldots ,T\;j=2,\ldots ,n, \end{array}$$

(4) $$\begin{array}{c} x_{\min}\leq x_{i}\leq \;x_{\max}\;i=1,\ldots ,T, \end{array}$$

(5) $$\begin{array}{c} x_{i}^{+}.x_{i}^{-}=0\;i=1,\ldots ,T, \end{array}$$

(6) $$\begin{array}{c} x_{i},\;x_{i}^{+}\;,\;x_{i}^{-},\;D,\;v_{ij},\geq 0\;m\;\geq 0,\text{ integer,} \end{array}$$

(7) $$\begin{array}{c} W,Z\in \left\{0,1\right\}. \end{array}$$

Equations (1) and (2) are objective functions of the proposed model. The first objective function minimizes the total cost of nurses. The first sentence of this function relates to nurses' fatigue reduction function at period *i*. The second and third sentences of the first objective function calculate the costs related to decisions about the increase or reduction in the number of nurses in each shift. Finally, the fourth and fifth sentences of the first objective function determine the number of shortages and surplus of nurses at period *i*. Equation (2) is the second objective function and minimizes the expected value of total fatigue for all nurses in all shifts. Appendix A provides some complementary relations and explanations about these objective functions.

Also, constraints of the proposed model have been formulated as equations (3)–(7). Constraint (3) shows nursing attendance virtual time at period *i*. Constraint (4) determines a lower bound and upper bound for nurse level changes at period *i*. Constraint (5) assures that in each period solely either nurse employment or nurse dismissal could occur. Finally, constraints (6) and (7) define the domains of the decision variables.

### 3.4. Linearization

The above-proposed model is nonlinear because of constraint (5). Therefore, before proceeding to the next stage, constraint (5) should be substituted with identical linear equations. To do so, equations (8)–(10) should be used:

(8) $$\begin{array}{c} x_{i}^{+}\leq P\cdot W, \end{array}$$

(9) $$\begin{array}{c} x_{i}^{-}\leq P\cdot Z, \end{array}$$

(10) $$\begin{array}{c} W+Z\leq 1. \end{array}$$

## 4. Solution Approach

Genetic Algorithm (GA) is one of the first Evolutionary Algorithms in which selection, crossover, and mutation are its main operators. The idea behind the GA originates from the Darwinian Theory of Evolutionary and, therefore, GA is categorized as a population-based algorithm. It can be said that the GA is a programming technique that uses genetic evolution as a pattern for solving problems. The GA algorithm starts with a random population. This population contains a set of solutions, which represent chromosomes of individuals. The next step is creating the second generation of the population based on selection processes, i.e., generation based on the selected characteristics by genetic operators. For each individual, a pair of parents is selected. In the selection stage, the most appropriate elements will be selected so that even the weakest elements have the chance to choose. This process prevents from nearing the local answer.

Generally, GA has a connectivity probability that is between 0.6 and 1, which indicates the probability of birth of a child, and the organisms combine with this possibility. The connection of two chromosomes creates the child, which is added to the next generation. This process is done to find the right candidates for the answer in the next generation. This process creates a new generation of chromosomes that are different compared with the previous generation. The whole process is repeated until the last stage [49].

In comparison with other optimization algorithms, GA has certain advantages. The most important one is that GA has a powerful ability to tackle complex problems and could be used for solving a wide variety of optimization problems with different objective functions (e.g., stationary or nonstationary objective functions, linear or nonlinear objective functions, etc.). Moreover, since “multiple off-springs in a population act like independent agents, the population (or any subgroup) can explore the search space in many directions simultaneously. This feature makes it ideal to parallelize the algorithms for implementation while different parameters and even different groups of encoded strings can be manipulated at the same time” [50].

Due to the aforementioned advantages, in this study, a hybrid GA algorithm is applied to solve the proposed NSP model.  Figure 1 shows the steps of the GA algorithm. Also, Appendix B provides more detail about the applied GA algorithm.

## 5. Computational Results

### 5.1. Model Validation

Prior to solving the model by using real data, to validate the accuracy of the proposed model, a test problem is generated randomly and a schedule for one week is provided.  Table 1 includes parameters for the test problem. All computations have been done within MATLAB software on a laptop with Intel Core i5, 2.5 GHz, and 4 GB of RAM.

The number of nurses is assumed to be five, and there are three shifts per day. Each nurse's salary per hour is also assumed to be 10 units per hour.

Table 2 shows the obtained schedule for a week for the test problem.

In Table 2, columns *x*_*i*_^+^ and *x*_*i*_^−^ show the required changes in the number of nurses so that the value in column *D* is affected by these changes in each row. Also, column F1 contains the imposed cots to the system by implementing the schedule whereas column F2 shows the fatigue of nurses.

### 5.2. Case Study

After validating the proposed model, we performed the model in a real case, a specific department of a hospital in Esfahan, Iran, where COVID-19 patients are hospitalized. Our purpose was to compare the scheduling obtained using the proposed model with those currently used in the considered department which have been computed manually by a person in the human resource department of the case study. Due to the nature of constraints in the NSP of the case study, the person who is responsible for providing the schedule, firstly, arranges an initial schedule that distributes all nurses within the days of a month. After that, she/he tries to rearrange the scheduling in order to also meet the fatigue of nurses as well. Accordingly, administrators of the department noted that the manual approach could be very time-consuming. In addition, some nurses were enjoying generous rest hours while most nurses were under high pressure. Thereby, administrators decided to automate the scheduling of this department. It led to the distribution of nurses within the shifts in a fair manner while the required time for providing a schedule was reduced significantly as well.

The department has 14 nurses, and working days are partitioned into three shifts: 8: 00 am-4: 00 pm, 4: 00 pm-12: 00 pm (0: 00 am), and 12: 00 pm-8: 00 am. Each nurse's salary per hour is 160000 IRR. It is worth mentioning that 1 EUR is equal to almost 46,292 IRR. Based on the salary, costs of employment, dismissal, shortage and, surplus are as follows:`

(11) $$\begin{array}{c} c_{1}=7*8*\text{nurse's salary per hour,}\\ c_{2}=22*8*\text{nurse's salary per hour,}\\ c_{3}=L_{i}*\text{nurse's salary per hour,}\\ c_{4}=2*L_{i}*\text{nurse's salary per hour.} \end{array}$$

The patient's arrival rate is based on the Poisson distribution and is *λ*_1_=2,  *λ*_2_=3, and *λ*_3_=3  in the first, second, and third shifts. The fatigue factor follows the Weibull distribution with parameters *ß* = 2 and *θ* = 500. Also, the parameters of the hybrid GA algorithm including the percentage of mutation, intersection percentage, and the number of repetitions are 0.1, 0.9, and 200, respectively. The model is solved within MATLAB software on a laptop with Intel Core i5, 2.5 GHz, and 4 GB of RAM.

The schedule for May which has been prepared manually and the schedule that has been prepared by hybrid GA have been compared in Table 3. In Table 3, column *D* depicts the order of each shift in each day. For instance, 6 3 3 on the 1st day of May states that, on the first day of May, the number of required nurses for the first, second, and third shifts is six, three, and three, respectively. In addition, columns *x*_*i*_^+^ and *x*_*i*_^−^ depict the level of changes required for each day regarding the last day. For example, on the 25th of May, one nurse should be added for a second shift whereas one nurse should be eliminated in the first shift compared with the 24^th^ of May. Therefore, the order of shifts on the 25th of May is 5 3 1 while on the 24^th^ of May the order was 6 2 1.

Column *m* presents the rest level at each shift. The value of 0 means that nurses will not be allowed to have further rest during their shift. In fact, all nurses have a break time generally in their shifts. If this usual break is the only break during the shift, *m* will give a value of 0. However, values of 1 and 2 for *m* state that nurses have one or two further breaks during their shift. Undoubtedly, the surplus break times reduce the fatigue of nurses dramatically.

Finally, columns F1 and F2 contain the value of costs and fatigue function in each day. It should be mentioned that F1 values have been divided into 1,000 for more convenience.

Figure 2 compares costs of manual scheduling and scheduling calculated by hybrid GA algorithm for all 31 days in May.

As Figure 2 illustrates, the costs of the department during one month according to manual scheduling are lower than those of the hybrid GA algorithm. However, this difference is not very significant, and Figure 3 clearly approves this matter. As it can be seen in Figure 3, the total costs of manual scheduling are 2,212,461,000 IRR while the total costs of scheduling which have been prepared by the proposed model and using the hybrid GA algorithm are 2,214,349,000 IRR. Therefore, the difference between costs is not higher than 2,000,000 IRR, and actually, this is not a considerable amount of money.

Figure 4 compares fatigue function in manual scheduling and hybrid GA scheduling.

Figure 4 clearly reveals that although the values of fatigue function in the second decade of May are almost identical in both hybrid GA scheduling and manual scheduling, the fatigue of nurses in hybrid GA scheduling is totally lower than that in manual scheduling.  Figure 5 which shows cumulative values of fatigue function for 31 days of May obviously approves this clime.

In addition, the required total time for providing a timetable by hybrid GA is considerably lower than the required total time for providing a timetable manually.  Figure 6 depicts this difference.

Figure 6 illustrates that scheduling of the department manually takes 66.67 minutes whereas the hybrid GA algorithm reduces the required time for scheduling dramatically so that it needs just 1.28 minutes for solving the proposed model and providing a timetable for the department.

## 6. Conclusion

Scheduling work shifts in many industry and service occupations directly affects the mental and physical health of employees. This matter can be more obvious in occupations like nursing where employees are usually working under high pressure and stress. Therefore, it would be better to consider employees' satisfaction and convenience in providing scheduling so that work hours impose lower pressure on them.

During the last months and due to the pandemic of COVID-19, physicians, nurses, and other persons in hospitals across the world are working under the highest pressure benevolently to suppress this insidious disease. This urgent situation can cause more fatigue for these persons, especially for nurses who are caring for COVID-19 patients 24 hours a day. Therefore, nurse scheduling should be modified with respect to this new situation.

In this paper, a mathematical model has been proposed to optimize the work shift of nurses considering human factors. To do so, according to experts' points of view, fatigue as the most important factor among human factors has been selected, and minimizing fatigue by creating different time intervals of rest during shift works has been addressed.

To solve the proposed model, a hybrid GA algorithm has been performed. In addition, to validate the efficiency of the proposed model, real data from the department of COVID-19 patients in one of the hospitals in Esfahan have been used where scheduling is currently determined manually. In fact, applying the proposed procedure of this paper, a timetable for all shifts of this department has been provided for May, and results have been compared with those currently used in the considered department and provided manually. Results approve that while the proposed approach imposes a little more cost to the department, it outperforms the current manual scheduling in both fatigue factor and time of providing a time table.

Apart from the lower required time for providing a timetable compared with the former manual approach, one of the main advantages of the proposed approach is eliminating personal tastes. It has been done because in the proposed approach, no one is involved in providing schedules, and the level of available resources is the only effective factor on the final schedule. To sum up, the proposed approach distributes nurses within the shifts in a fair manner considering the least fatigue while the required time for providing a schedule is significantly lower than the manual approach as well. However, another strength of our proposed approach is its generalizability. In other words, due to the structure of formulation, the proposed model could be used in either other healthcare departments or other continuous systems where a schedule for different shifts is required. In all of these settings, the model could distribute nurses/workforces within different shifts fairly considering least fatigue.

In future research, our model can be developed by considering other human factors such as rewards, motivation, and loyalty. Also, developing other heuristic and metaheuristic techniques would be an interesting direction for future research.

## Figures and Tables

**Figure 1:** Steps of the GA algorithm.

**Figure 2:** Comparison of the cost function.

**Figure 3:** Cumulative values of the cost function.

**Figure 4:** Comparison of fatigue function.

**Figure 5:** Cumulative values of fatigue function.

**Figure 6:** Required time for providing a schedule.

**Table 1:** Input parameters of test problem.

Parameters	Values
*c*_1_, *c*_2_, *c*_3_, *c*_4_	Uniform (1, 10)
*λ*	1
Β	1
*θ*	20

**Table 2:** Schedule for the test problem.

Day (i)	*x*_*i*_^+^	*x*_*i*_^−^	m	D	F1 (cost)	F2 (fatigue)
1	0 0 0	0 0 0	0 0 0	2 1 1	2,156	0.0386
2	0 0 1	0 0 0	0 0 1	2 1 2	2,798	0.0369
3	0 1 0	0 0 1	2 1 0	2 2 1	2,604	0.0358
4	0 0 0	0 1 0	2 0 0	2 1 1	2,309	0.0258
5	0 0 0	0 0 0	1 0 0	2 1 1	2,255	0.0344
6	0 0 1	0 0 0	1 0 1	2 1 2	2,885	0.0361
7	0 1 0	0 0 1	1 1 0	2 2 1	2,515	0.029

**Table 3:** Scheduling of May provided by hybrid GA and manually.

Day (i)	Manually (hospital)						Hybrid GA					
	*x*_*i*_^+^	*x*_*i*_^−^	m	D	F1 (cost)	F_2_ (fatigue)	*x*_*i*_^+^	*x*_*i*_^−^	m	D	F1 (cost)	F2 (fatigue)
1	0 0 0	0 0 0	0 0 0	6 3 3	71,481	0.0591	0 0 0	0 0 0	0 0 0	6 3 3	71,481	0.0591
2	0 0 0	0 0 0	0 0 1	6 3 3	73,123	0.0574	0 0 0	0 0 0	0 0 1	6 3 3	73,123	0.0574
3	0 0 0	0 0 0	0 0 2	6 3 3	76,729	0.0563	0 0 0	0 0 0	0 0 2	6 3 3	76,729	0.0563
4	0 0 0	0 0 0	1 0 0	6 3 3	74,992	0.0581	0 1 0	1 0 0	2 0 2	5 4 3	75,834	0.0463
5	0 0 0	0 0 0	1 0 1	6 3 3	77,440	0.0549	1 0 0	0 1 0	1 0 1	6 3 3	77,440	0.0549
6	0 0 0	0 0 0	1 0 2	6 3 3	78,070	0.0535	0 0 0	1 0 0	2 0 2	5 3 3	73,810	0.0566
7	0 0 0	0 0 0	1 1 1	6 3 3	81,770	0.0532	0 0 0	0 0 1	2 0 2	5 3 2	69,410	0.0495
8	0 0 0	0 0 0	1 1 2	6 3 3	89,200	0.0498	0 0 0	0 0 0	2 1 2	5 3 2	71,618	0.0448
9	0 0 0	0 0 0	2 0 1	6 3 3	79,250	0.0541	1 0 1	0 0 0	2 0 1	6 3 3	79,250	0.0541
10	0 0 0	0 0 0	2 0 2	6 3 3	83,880	0.0526	0 0 0	1 0 1	2 2 2	5 3 2	72,431	0.0507
11	0 0 0	0 0 0	1 1 2	6 3 3	89,200	0.0498	0 1 1	0 0 0	2 1 2	5 4 3	91,012	0.0455
12	0 0 0	0 0 0	2 2 2	6 3 3	92,310	0.0479	1 0 0	0 1 0	2 2 2	6 3 3	92,310	0.0479
13	0 0 0	0 0 0	1 0 2	6 3 3	78,070	0.0535	0 0 0	0 0 0	1 0 2	6 3 3	78,070	0.0535
14	0 0 0	0 0 0	2 2 2	6 3 3	92,310	0.0479	0 0 0	0 0 0	2 2 2	6 3 3	92,310	0.0479
15	0 0 0	0 0 0	2 0 0	6 3 3	74,235	0.0588	0 0 0	0 0 0	2 0 0	6 3 3	74,235	0.0588
16	0 0 0	0 0 0	1 0 1	6 3 3	77,440	0.0549	0 0 0	1 0 0	2 1 1	5 3 3	74,142	0.0571
17	0 0 0	0 0 0	2 0 2	6 3 3	83,880	0.0526	1 0 0	0 0 0	2 0 2	6 3 3	83,880	0.0526
18	0 0 0	0 0 1	2 0 2	6 3 2	68,300	0.0598	0 0 0	0 0 1	2 0 2	6 3 2	68,300	0.0598
19	0 0 0	0 0 0	2 1 2	6 3 2	70,173	0.0576	0 0 0	0 0 0	2 1 2	6 3 2	70,173	0.0576
20	0 0 0	0 0 0	2 2 2	6 3 2	72,345	0.0561	0 0 0	0 0 0	2 2 2	6 3 2	72,345	0.0561
21	0 0 0	0 0 1	2 0 2	6 3 1	60,900	0.0661	0 0 0	1 0 0	2 2 2	5 3 2	63,476	0.0609
22	0 0 0	0 0 0	1 1 2	6 3 1	62,200	0.0649	0 0 0	0 0 0	2 2 0	5 3 2	60,150	0.0637
23	0 0 0	0 0 0	1 1 0	6 3 1	59,145	0.0674	0 1 1	0 0 0	2 1 1	5 4 3	63,182	0.0528
24	0 0 0	0 1 0	1 1 1	6 2 1	51,165	0.0801	0 0 0	1 2 1	2 2 2	4 2 2	52,750	0.0746
25	0 1 0	1 0 0	2 2 2	5 3 1	54,100	0.0681	1 1 0	0 0 1	2 2 2	5 3 1	54,100	0.0681
26	0 0 1	0 1 0	2 2 2	5 2 2	56,108	0.0768	0 0 1	0 1 0	2 2 2	5 2 2	56,108	0.0768
27	1 1 0	0 0 0	2 2 2	6 3 2	72,345	0.0561	0 1 1	0 0 0	1 1 1	5 3 3	71,230	0.0574
28	0 0 0	2 1 0	2 2 2	4 2 2	52,215	0.0795	1 0 0	0 1 1	2 2 2	6 2 2	58,900	0.0646
29	0 0 1	0 0 0	2 2 2	4 2 3	54,000	0.0835	0 1 1	0 0 0	2 1 2	6 3 3	71,700	0.0513
30	1 1 0	0 0 2	2 2 2	5 3 1	54,100	0.0681	0 0 0	1 1 0	2 1 2	5 2 3	55,700	0.0662
31	0 0 1	1 1 0	0 0 0	4 2 2	51,985	0.0919	1 0 0	0 0 0	2 1 2	6 2 3	69,150	0.0598

## Data Availability

The data used to support the findings of this study are available from the corresponding author upon request.

## Appendix

### A. Complementary Relations

As mentioned in Section 3.3, the first objective function minimizes the total cost of nurses. The first sentence of this function relates to nurses' fatigue reduction function at period *i* which is calculated based on equation (A.1):

(A.1) $$\begin{array}{c} c_{PM}\left(i\right)=m\cdot \Delta_{i}.c_{5}.a^{m.\gamma },\;i=1,\ldots ,T, \end{array}$$

The second and third sentences of the first objective function calculate the costs related to decisions about the increase or reduction in the number of nurses in each shift. In other words, *x*_*i*_^+^ depicts the number of employed nurses while *x*_*i*_^−^ shows the number of dismissed nurses at period *i*. Finally, the fourth and fifth sentences of the first objective function determine the number of shortages and surplus of nurses at period *i*. On the one hand, when demand is higher than the number of nurses (D >  *x*_*i* _), the cost of shortage could be computed as follows:

(A.2) $$\begin{array}{c} c_{3}\overset{T}{\underset{i=1}{\sum }}\left(D-x_{i}\right)f\left(d\right). \end{array}$$

On the other hand, when demand is less than the number of nurses (*D* ≤  *x*_*i* _), the cost of the surplus could be computed as follows:

(A.3) $$\begin{array}{c} c_{4}\sum_{i=1}^{T}\left(D-x_{i}\right)f\left(d\right)\;D\leq \;x_{i\;}. \end{array}$$

It should be noted that *x*_*i*_ is computed based on equation (A.4) and (A.5):

(A.4) $$\begin{array}{c} x_{i}=x_{i-1}+x_{i}^{+}-x_{i}^{-}\;i=1,\ldots ,T. \end{array}$$

Since *D* is a Poisson random variable, *f*(*d*) in equations (A.2) and (A.3) is a Poisson distribution function. Therefore, equations (A.2) and (A.3) should be rewritten as the following equations:

(A.5) $$\begin{array}{c} c_{3}\sum_{i=1}^{T}\left(D-x_{i}\right)\frac{e^{-\lambda t}\cdot \lambda t^{D}}{D!}\;\;\;D>\;x_{i\;},\\ c_{4}\sum_{i=1}^{T}\left(D-x_{i}\right)\frac{e^{-\lambda t}\cdot \lambda t^{D}}{D!}\;\;D\leq \;x_{i\;}. \end{array}$$

Moreover, as mentioned in Section 3.3, the proposed model has a second objective function which minimizes the expected value of total fatigue for all nurses in all shifts. In the current objective function, there are some values that will be calculated using the following equations:

(A.6) $$\begin{array}{c} v_{ij}\left(t\right)=\left\{\begin{array}{cc} t_{i} & t_{i}<\tau_{i1}\;\;i=1,\ldots ,T\\ v_{ij-1}+t+\tau_{ij-1} & \tau_{ij-1}\leq t<\tau_{ij\;}\;\;j=2,\ldots ,n \end{array}\right.,\\ F\left(v_{ij}\left(t\right)\right)=\left\{\begin{array}{cc} F\left(t\right) & t_{i}<\tau_{i1},\;F\;\left(t\right)<b\;i=1,\ldots ,T\\ F\left(v_{ij-1}+t-\tau_{ij-1}\right) & \tau_{ij-1}\leq t<\tau_{ij,\;F\;\left(t\right)<b\;}\;i=1,\ldots ,T,\;j=2,\ldots ,n\\ 0 & \;F\;\left(t\right)\geq b. \end{array}\right., \end{array}$$

### B. Steps of the Hybrid GA Algorithm

#### 1) Generating Initial Answer

Since there are four variables including  *x*_*i*_^+^, *x*_*i*_^−^,  *m* ,  *D* and three shifts, all feasible solutions will be revealed in the form of a 4 × 3 matrix. A feasible answer can be found as follows:

(B.1) $$\begin{array}{c} \begin{array}{cccc} x_{i}^{+}⟶ & 0 & 1 & 0\\ x_{i}^{-}⟶ & 2 & 0 & 1\\ m⟶ & 1 & 2 & 1\\ D⟶ & 4 & 4 & 2 \end{array}. \end{array}$$

An initial answer will be generated randomly. For this purpose, one of the first or second rows is selected randomly. To fill the first column, a random number between [*x*_ min_, *x*_ max _] is selected. If the selected number is greater than zero, we will write a zero in the next row while if the selected number is zero, a random number in the interval [*x*_ min_, *x*_ max _] will be selected for another row. The same procedure will be employed for the second and third columns as well. In the third row, a random number in the interval [*x*_ min_, *x*_ max _] opts for the first to third columns respectively.

#### 2) Fitness Function

Suppose *f*_1_=*c*_1_∑_*i*=1_^*T*^*x*_*i*_^+^ and *f*_2_=*c*_2_∑_*i*=1_^*T*^*x*_*i*_^−^. The fitness function is calculated according to these functions and will put in the Pareto set.

#### 3) Generating New Answer Based on Different Neighborhood Structures

  The first neighborhood structure is as follows:
  Between the first and second rows, one of them is chosen randomly. Suppose that *i* represents the selected row. Now a random column like *j* is chosen randomly. If *x*_*ij*_+1 ≤ *x*_max_, then *x*_*ij*_+1⟶*x*_*ij*_ and the value of column *j* in the next row is zero.
  The second neighborhood structure:
  Between the first and second rows, one of them is chosen randomly. Suppose that *i* represents the selected row. Now, a random column like *j* is chosen randomly. If *x*_*ij*_ − 1 ≥ *x*_min_, then *x*_*ij*_ − 1⟶*x*_*ij*_.
  The third neighborhood structure:
  In the third row, a column *j* is chosen randomly. If *m*_*j*_+1 ≤ *m*_max_, then, *m*_*j*_+1⟶*m*_*j*_.
  The fourth neighborhood structure:
  In the third row, a column *j* is chosen randomly. If *m*_*j*_ − 1 ≥ *m*_min_, then, *m*_*j*_ − 1⟶*m*_*j*_.
  The algorithm starts with the first neighborhood structure. The answer is added to the Pareto set; therefore, the current neighborhood structure remained. Otherwise, go to the next neighborhoods' structure. It should be mentioned that once the newly generated answer is entered into the Pareto set, the algorithm starts with the first neighborhood structure again. In this situation, the algorithm replicates the search process for *m* times.

#### 4) Evaluating the New Generated Answer

  In the evaluation stage of the new generated answer, one of the following states should occur:
  First state
  If *f*_1_ ,  *f*_2_  for the new answers, in all answers of the dominant set, are worse, or one of them is worse and another is equal, it is not allowed to enter the dominant answer set.
  Second state
  The new answer is better than k answers of the dominant answer set. So, the new answer is added to the dominant set, and *k* nondominant answers will be eliminated.
  Third state
  The new answer is not better than any answers of the dominant answer set. Meanwhile, if one of the functions *f*_1_ or *f*_2_ is superior to all answers of the dominant answer set, it will enter into the Pareto set. However, other answers will remain in the dominant answer as well.

#### 5) Replicating Algorithm

  Steps 1 to 3 are replicated for *m* times.
